The article "A Novel Adaptive Affective Cognition Analysis Model for College Students Using a Deep Convolution Neural Network and Deep Features" was published in 2022. Journal: Comput Intell Neurosci.

# A Novel Adaptive Affective Cognition Analysis Model for College Students Using a Deep Convolution Neural Network and Deep Features

**DOI:** 10.1155/2022/2114114

**Published:** 2022-08-27

**Authors:** Huali Feng

**Affiliations:** Data and Information Center, Wuxi Vocational Institute of Commerce, Wuxi 214153, Jiangsu, China

## Abstract

Currently, under the impact of the COVID-19, college students are facing increasingly elevated employment pressure and higher education pressure. This can easily cause a huge psychological burden on them, causing affective cognition problems such as anxiety and depression. In the long run, this is not conducive to students' physical and mental health, nor is it conducive to the healthy development of the school and even the whole society. Therefore, it is imperative to build a novel adaptive affective cognition analysis model for college students. In particular, in the context of smart cities and smart China, many universities have opened the smart campus mode, which provides a huge data resource for our research. Due to problems of the low real-time evaluation and single data source in traditional questionnaire evaluation methods, evaluation errors are prone to occur, which in turn interferes with subsequent treatment. Therefore, for the purpose of alleviating the above deficiencies and improving the efficiency and accuracy of the affective cognition analysis model of college students, this paper studies the adaptive affective cognition analysis method of college students on basis of deep learning. First, because students' psychological problems are often not sudden, on the contrary, most of these abnormalities will leave traces in their daily activities. Therefore, this paper constructs a multisource dataset with the access control data, network data, and learning data collected from the smart campus platform to describe the affective cognition status of students. Second, the multisource dataset is divided into two categories: image and text, and the CNN model is introduced to mine the psychological characteristics of college students, so as to provide a reference for the subsequent affective cognition state assessment. Finally, simulation tests are developed to confirm the viability of the technique suggested in this research. The experiments demonstrate that the accuracy of the assessment model is significantly increased because it can fully reflect the heterogeneity and comprehensiveness of the data. This also highlights that the new method has a wide range of potential applications in the modern campus setting and is also helpful in fostering the accuracy and depth of college students' work on their affective cognition.

The article "A Novel Adaptive Affective Cognition Analysis Model for College Students Using a Deep Convolution Neural Network and Deep Features" was published in 2022. Journal: Comput Intell Neurosci.

## 1. Introduction

Because life is moving at an increasingly rapid speed, people's mental health is deteriorating, and more and more people are facing depression, autism, insomnia, and other psychological problems [1]. Simultaneously, under the impact of the COVID-19, college students are facing increasing pressure for higher education and employment, leading to an increasing number of college students suffering from different degrees of depression and anxiety disorders. In other words, various mental health problems have slowly penetrated into all aspects of college students' daily life, so that their bodies and psyches are suffering from different degrees of destruction [2]. Currently, according to reports, there have been an increasing number of extremely dangerous occurrences involving college students brought on by psychological issues, such as suicide, self-harm, and fights and brawls occur frequently [3]. Therefore, paying attention to the college students' affective cognition and studying a set of scientific and effective affective cognition analysis methods is one of the problems that colleges and universities urgently need to solve. This not only helps ensure the safety of students' lives during school, but also helps them complete their studies smoothly. It can also provide support for the promotion of smart mental health education in universities.

With the aid of various digital and intelligent technologies, universities are gradually transitioning to the age of the smart campus. Relying on these technologies, a smart campus is an effort to create an intelligent teaching environment, intelligent management mode, and digital teaching resources to form a new ecology of learner-centered education and teaching, which is an inevitable trend for digital school reform [4, 5]. In the intelligent campus environment, students' life and learning data will be recorded into various management systems. These massive data contain a huge amount of information and provide a better opportunity to grasp their psychological and affective cognition state. It can be said that the flourishing development of smart campus will open a new door for the study of college students' affective cognition. At the present stage, related research still rely on the modes of questionnaires and structured interviews, which have many shortcomings, such as the insufficient amount of data, single data source, easy to conceal the truth and mislead the assessment results, lack of timeliness of assessment results, and passive assessment work [6]. In response to the drawbacks of traditional assessment methods, some scholars have tried to do some improvement work. They used social network data in affective cognition assessment studies and realized automatic affective cognition analysis with the help of trained models, and achieved relatively satisfactory assessment results [7]. However, the shortcoming is that these methods still face problems such as difficulties in collecting data on network behaviors and incomplete information on single-modal data, which make it difficult to judge the affective cognition status of the assessed person accurately and comprehensively.

The article "A Novel Adaptive Affective Cognition Analysis Model for College Students Using a Deep Convolution Neural Network and Deep Features" was published in 2022. Journal: Comput Intell Neurosci.

Technology empowers education, and the ability to autonomously assess students' affective cognition state has been made available by the deep learning technology's quick development. After years of building information application systems, schools have accumulated massive amounts of data on teaching, consumption, and student behavior. With the continuous accumulation of these data, if the sentiment tendencies of students can be mined from these multisource data, it will help to know the affective cognition status of students more accurately. If the manual labeling method is still used to deal with such a large amount of data, it is indeed labor and time intensive. Moreover, the accuracy of the information obtained is low. In view of this, for the purpose of improving the accuracy and effectiveness of college students' affective cognition analysis model, it is very important to use deep learning architecture to classify and predict related data in practical applications. Deep learning has been one of the key directions of academic research recently. Additionally, it has made significant strides in the research of college students' affective cognition [8–10]. Many scholars have proposed to use deep neural network models such as CNN [11] and Bi-LSTM [12] to analyze and train the influencing factors affecting students' affective cognition problems and establish analytical models to classify and predict students' affective cognition problems. In addition, the literature [13] and the literature [14] applied the massive data recorded by the relevant systems on campus to mine the behavioral data related to students' affective cognition. Meanwhile, artificial intelligence algorithms are used to intelligently identify students' abnormal behavior and construct early warning models. The affective cognition problems of college students are detected in time and precise psychological counseling is provided for them.

The above research shows that deep learning technology provides a new perspective for students' affective cognition work to take the road of precision and wisdom. In view of this, this study closely combines college students' affective cognition work with the construction work of smart campus. In the research, the advantages of deep learning technology are fully utilized and based on the multisource data such as access control data, learning behavior data, and network data recorded in the smart campus platform, an adaptive affective cognition analysis model for college students is constructed for the purpose *f* improving the effectiveness and accuracy of psychological state assessment of college students. The research work mainly includes: first, carefully studying relevant domestic and foreign literature, closely combining the multisource data recorded in the smart campus environment, including access control data, learning behavior data, and network data, and building a multisource dataset. Second, on the premise of information security, the multisource data set is divided into two categories: image and text, and the CNN model is introduced to process and analyze these data. In this way, the hidden affective cognition problems of students in these data can be excavated, and the mental health status of college students can be accurately identified. Finally, simulation tests are developed to confirm the viability of the technique suggested in this research. The experiments demonstrate that the novel technique has a higher identification accuracy when assessing the affective cognition state of college students compared with the data of a single modality. It can accurately grasp students' mental health status and has broad application prospects in the smart campus environment.

The article "A Novel Adaptive Affective Cognition Analysis Model for College Students Using a Deep Convolution Neural Network and Deep Features" was published in 2022. Journal: Comput Intell Neurosci.

## 2. Related Theory

### 2.1. Artificial Intelligence and Deep Learning

Artificial intelligence (referred as “AI”) allows machines to simulate or realize the process of human learning behavior by computing and analyzing some human thinking, consciousness, and behavior with the help of mathematical tools [15]. Currently, as new technologies and industries arise, AI has been given more expectations and heavy responsibilities. At present, it has made great achievements in iris recognition, face recognition, intelligent search, and other fields [16, 17]. The scope of artificial intelligence is shown in Figure 1.

As one of the representative technologies in the field of AI, machine learning studies human learning behavior and is the core of artificial intelligence. It mainly refers to the computer through the automatic analysis of data, facts, or its own experience, and then comprehensively acquire new knowledge or skills, so that the computer can have the ability to automatically learn specific knowledge and skills, and establish a task-oriented learning system with specific applications [18]. It can be said that it is the fundamental way to make computers intelligent. As a subset of machine learning, deep learning aims to achieve the universalization of artificial intelligence. Deep learning was first proposed by Hinton et al. to study the optimal representation of information and its acquisition method. In the case of neural networks or belief networks, it is the process of machine learning of the mapping between inputs and outputs based on deep structures or network representations [19]. Currently, deep learning is a hold expression for a group of pattern recognition techniques. Convolutional neural networks, multilayer neuron-based autoencoder neural networks, and deep belief networks are basically the three forms of convolutional neural networks that are relevant to the specific study material. Because deep learning makes it possible for machines to accurately simulate some aspects of human society and is useful for many complex recognition patterns, it has greatly contributed to the development of related fields such as artificial intelligence. In the last 30 years or so, research on this topic has attracted the close attention of many scholars, and significant progress has been made in areas such as natural language processing [20], image processing [21], data mining [22], and machine translation [23].  Figure 2 shows the difference in principle between deep learning and several other machine learning techniques.

The article "A Novel Adaptive Affective Cognition Analysis Model for College Students Using a Deep Convolution Neural Network and Deep Features" was published in 2022. Journal: Comput Intell Neurosci.

### 2.2. Deep Neural Network

The specific process of deep learning can be briefly described as: train a multilayer neural network to mine the inherent laws and connections of the given sample data. Extract and analyze the characteristic information of samples, such as images, texts, and sounds. Process data information and issue instructions to control the behavior of the machine, so that the machine has the capabilities of learning, analysis, recognition, and processing similar to humans. As a representative of deep learning technology, Deep Neural Network (referred as DNN) has received wide attention since its introduction. Based on the traditional neural network, it expands the hidden layer to multiple layers, which can better deal with the problem of the network in dealing with complex functions, and greatly improve the performance of the model [24]. The network structure of DNN is shown in Figure 3.

It has been shown that the training process of traditional neural networks can be essentially divided into two key steps forward computation and backward propagation. And through repeated loops, iterates continuously until the final convergence condition is reached, the model training ends, and the training results are output. The difference between DNN and traditional neural networks is that the former introduces several hidden network learning units between the input layer and the output layer, thereby greatly improving the training efficiency of the model and the ability to process complex data.

The article "A Novel Adaptive Affective Cognition Analysis Model for College Students Using a Deep Convolution Neural Network and Deep Features" was published in 2022. Journal: Comput Intell Neurosci.

## 3. An Adaptive Affective Cognition Analysis Model Based on Deep Learning

The affective cognition analysis model for college students based on deep learning covers the following two core steps: (1) On the basis of the smart campus platform, we collect multiple sources of student behavior data to build an adaptive affective cognition analysis system for college students, including access control data, learning data and network data, so as to more comprehensively portray the psychological indicators of students. (2) The multisource data are divided into two categories: image and text, and then the CNN model is applied to mine the students' emotions and psychological changes hidden in these data, so as to accurately assess the students' affective cognition level.  Figure 4 illustrates the framework of the assessment model based on multisource data.

As shown in Figure 4, the general process of our research model consists of three main parts, which are sentiment calculation based on text data, sentiment calculation based on image data, and sentiment calculation of image-text fusion data. First, in this study, we collected three types of data sources access control data, learning data, and network data and preprocessed these multisource data. Second, we divide the collected multisource data into two categories image and text and then compute the affective values using CNN models, respectively. Finally, in the model training and recognition stage, the text and image affective values are fused and calculated using the maximum value rule. At the same time, it is compared with the constructed affective cognition analysis model, and finally, the mental health level is output.

### 3.1. Multisource Data

With the rise of smart campuses, a large amount of student behavior data has been preserved, which records the bits and pieces of students' study and life during school. These data are both in the form of images and texts, which can feedback a student's psychological changes in a certain period of time from different perspectives. By mining and analyzing these data, it helps to assess students' current affective cognition conditions more comprehensively and systematically. Therefore, collecting data that can accurately represent the features of college students' affective cognition is a necessary first step in analyzing their mental health.  Figure 5 depicts the complete multisource data system.

As shown in Figure 5, our research focuses on the following data sources:

The article "A Novel Adaptive Affective Cognition Analysis Model for College Students Using a Deep Convolution Neural Network and Deep Features" was published in 2022. Journal: Comput Intell Neurosci.

### 3.2. Network Data

Research has shown that there is a relationship between online behavior and psychological traits such as personality, mood, and depression. Using students' online data can graphically portray their psychological and affective cognition characteristics. From a psychological point of view, the information posted by college students on forums, the content of social chats, the music playlists they listen to, and the students' online active time are all affected by the students' affective cognition. Web logs record these data of students' online characteristics, and how to dig out students' affective cognition characteristics from these records is the problem we want to solve.

### 3.3. Earning Behavior Data

In the field of education research, significant negative correlations were found between mild, moderate, and severe depression and academic performance. The student's learning behavior data reflect the student's past learning state and process. Introducing these data can be helpful to our research. In a smart campus environment, cameras in the classroom can be utilized to capture data on students' learning behaviors in the classroom, such as sleeping in class, playing with cell phones, depressed mood, and other abnormal behaviors.

### 3.4. Access Control Data

Similarly, some surveys found that there is a strong link between the level of interpersonal relationships and the level of affective cognition. As a result, we can identify students who have mental health issues by extracting indicators that reflect students' social relationships. Access control data show more than just the timing of students entering and exiting the dormitory. Often, using the image data recorded by the access control system of students entering and leaving the dormitory with their friends or roommates, mining in this direction may also reveal information of interest to us such as their interpersonal relationships. Therefore, our research also benefits from the mining of students' social relationship features using access control data.

In summary, with the help of the data center in the smart campus, the multisource data that may contain the psychological and affective cognition characteristics of students can be collected and integrated to form a 360-degree portrait of students. Based on the multisource data, we can establish an affective cognition analysis model for college students to detect problems in time and provide proactive early warning to teachers and administrators, so as to realize the development of students' psychological problems from “passive management” to “active prevention”.

### 3.5. CNN Network Model

#### 3.5.1. Model Training Based on Text Data

The CNN training model based on text data applied in this study is shown in Figure 6. It contains several convolutional layers, pooling layers, and a fully connected layers.

The article "A Novel Adaptive Affective Cognition Analysis Model for College Students Using a Deep Convolution Neural Network and Deep Features" was published in 2022. Journal: Comput Intell Neurosci.

First, in the input layer, the collected text data needs to be word partitioned. That is, the input text content is segmented into word vectors of length *N* using Word2Vec technique [25], as shown in formula (1).

(1) $$\begin{array}{c} T=\left[t_{1},t_{2},\ldots ,t_{N}\right],\;t_{i}\in R^{l\times h}. \end{array}$$

Then, in the convolution layer, the word vectors in formula (1) are further processed one by one using the convolution operation, and the detailed process is illustrated in formula (2) and formula (3).

(2) $$\begin{array}{c} \langle t_{0:k-1},t_{1:k},\ldots ,t_{N-k+1:N}\rangle , \end{array}$$

(3) $$\begin{array}{c} f_{j}=\partial \left(\varphi \left(\omega •T_{i-j+k-1}+\beta \right)\right), \end{array}$$

where *φ* represents the convolution kernel function and *f*_*j*_ indicates the eigenvalues obtained after convolution.

The convolution result is further de-linearized, and the link requires the introduction of an activation function, as shown in formula (4). The processed structure is then stitched to obtain the feature matrix *F*, as shown in formula (5).

(4) $$\begin{array}{c} \delta \left(t\right)=\frac{1}{1+e^{-t}}, \end{array}$$

(5) $$\begin{array}{c} F=f_{1}⊕f_{2}⊕\cdots ⊕f_{N-k+1}. \end{array}$$

In the pooling layer, this study utilizes the maximum pooling method to reduce the dimensionality of the feature matrix obtained from the convolutional layer to prevent the overfitting problem and to increase the operational effectiveness of the network simultaneously. The method is shown in formula (6).

(6) $$\begin{array}{c} F=\left\{\max\left(f_{1}\right),\max\left(f_{2}\right),\ldots ,\max\left(f_{N-k+1}\right)\right\}. \end{array}$$

The fully connected layer further processes the features extracted by the pooling layer to obtain the final feature vector, as shown in formula (7).

(7) $$\begin{array}{c} H=\sum_{i=1}^{N-k+1}\left(\omega •F_{i}+\beta_{i}\right). \end{array}$$

Finally, in the output layer, the final feature vector is predicted for classification using the softmax function and the computed results are output. The detailed process is shown in formula (8) and formula (9).

(8) $$\begin{array}{c} y=\text{soft }\max\left(V•H+\lambda \right), \end{array}$$

(9) $$\begin{array}{c} \text{soft }\max\left(t\right)=\frac{e^{t}}{\sum_{k=1}^{K}e^{t}}. \end{array}$$

#### 3.5.2. Model Training Based on Image Data

As an important supplement to textual information, accurate identification of the psychological and affective cognition characteristics of students embedded in image data is also very important. Image-based affective computing is a challenging visual problem. Only by learning a large number of parameters and effective features, the CNN model can precisely calculate the psychological sentiment contained in image data. This study utilizes the VGG16 convolutional base as a pretrained model for image affective tendencies computing to learn general feature representations and abstract feature representations for images. Meanwhile, the original dense connection layer settings are changed to suit the task of image affective computing. This can significantly increase the CNN model's applicability and reduce the chance of overfitting during model training.

The article "A Novel Adaptive Affective Cognition Analysis Model for College Students Using a Deep Convolution Neural Network and Deep Features" was published in 2022. Journal: Comput Intell Neurosci.

We initially utilize the capabilities of several convolutional layers in the VGG16 convolutional base to learn the sentiment representation of images during the training of the CNN model. Then, the extracted image affective features are integrated and classified by the dense connection layer. Finally, the affective tendency value of the image is output.

#### 3.5.3. Computation of Multisource Data Using the Maximum Value Rule

Finally, this paper adopts the maximum value rule to compute the affective tendency value of text and image data in order to precisely analyze the level of college students' affective cognition. In this way, it fully takes into account the affective characteristics of these two types of data. Formulas (10) and (11) illustrate the precise computation procedure.

(10) $$\begin{array}{c} Y_{j}^{\prime }=\underset{i}{\max}\left(Y_{ij}\left(N\right),\;i=1,2\text{, }j=1,2\right., \end{array}$$

(11) $$\begin{array}{c} Y_{j}\left(N\right)=\frac{Y_{j}^{\prime }\left(N\right)}{\sum_{j}Y_{j}^{\prime }\left(N\right)}, \end{array}$$

where *i* and *j* indicate the number of classifiers and categories, respectively, and *Y*_*j*_ (*N*) represents the probability value of the *j*th sentiment category.

## 4. Experimental Test

### 4.1. Data Set and Data Processing

To evaluate how well the method put forward in this work performs when used in practice, we recruited subjects from college students in a university in Wuxi to design simulation tests. Based on the principle of voluntary enrollment, a total of 200 subjects were recruited for the experiment. They were then given depression self-assessment questionnaires designed according to the CES-D scale. Then, the collected questionnaire data was cleaned, and the affective cognition grades of the experimental subjects were marked according to the scores of the questionnaires, which were divided into three categories: healthy, possible depression, and existing depression. The distribution of the three cases was 135 (67.5%), 42 (21%), and 23 (11.5%). In addition, with the consent of 200 subjects, a confidentiality agreement was signed with them to collect the behavioral data of the subjects from the school's smart platform, including access control data, learning data, and Internet access data, to construct a multisource data set. What's more, experts in related fields were invited to label these multisource data according to their emotional disposition and classify them into two categories: positive emotions and negative emotions. Thus, a joint annotation dataset for psychological assessment is formed, and Table 1 illustrates the detailed data distribution.

The article "A Novel Adaptive Affective Cognition Analysis Model for College Students Using a Deep Convolution Neural Network and Deep Features" was published in 2022. Journal: Comput Intell Neurosci.

Whether it is the data of students' affective cognition level collected in the form of questionnaires or the multisource data about students' behavior collected by the smart platform, they cannot be directly used in the model for psychological assessment. Therefore, data cleaning needs to be performed on these raw data, including questionnaire data processing and text and image data processing in multisource data. Finally, the cleaned data are preprocessed, i.e., they are transformed into data types that can be recognized by the CNN model. For example, for text data, the irrelevant symbols are removed and the fonts are converted. For image data, format conversion, size adjustment, and normalization are performed.

## 5. Results and Analysis

In the simulation experiments, three representative evaluation metrics are utilized to verify the evaluation effect of the model, which are Precision, Recall, and F1-Measure.

First, to verify the effectiveness of the proposed method in the application of affective cognition assessment for college students in this paper, the following simulation experiments are designed: (1) Calculate the assessment results based on text data using CNN model. (2) Calculate the assessment results based on image data using CNN model. (3) Calculate the assessment results based on the fusion of text and image using the maximum rule.  Figure 7 illustrates the assessment results for different data forms.

Observing Figure 7, we can conclude the following:

1. Overall, the proposed method of fusing multisource data in this paper achieves relatively satisfactory assessment results in all three evaluation indexes, and the results reach more than 85%. This indicates that, due to the utilization of the maximum value rule calculation in the new method, the advantages of text data and image data can be fully utilized, allowing the two to form a complementary relationship, thus overcoming the drawback of single data in the traditional assessment method and greatly improving the assessment accuracy of the model.
2. Second, among the assessment results of three different data forms, the assessment result based on fusion data has the best performance, which is significantly better than that of text data and image data. Moreover, the assessment results based on text data are also more desirable than those based on image data. However, despite this, the influence of image data on the assessment results cannot be ignored. On the contrary, because image data can be a key supplement to text data, it can sometimes express students' emotions and feelings more directly and graphically, and even convey some mental states that cannot be depicted by textual language. In this study, we integrate them with text data to fully exploit the benefits of various data types and to produce a more thorough assessment and analysis of students' affective cognition conditions.

The article "A Novel Adaptive Affective Cognition Analysis Model for College Students Using a Deep Convolution Neural Network and Deep Features" was published in 2022. Journal: Comput Intell Neurosci.

In addition, to further verify the feasibility and usefulness of our research model in real life, the scores based on the questionnaire scales were compared with the assessment results of the model to produce the final mental health assessment accuracy.  Figure 8 displays the detailed assessment results.

The results in Figure 8 reveal that among the assessment results of the three mental health levels, the recognition accuracy for the health level is the highest, reaching 91.6%. Followed by the existing depression level, its recognition accuracy was 85.3%. The lowest accuracy was obtained for the possible depression level, which was 80.6%. The difference between the assessment accuracy of the health level and the assessment accuracy of the possible depression level is nearly 10%, and the gap is relatively obvious. The reason is that, whether students in the healthy level or in the existing depression level, their affective cognition in these two states is in a relatively stable positive state or negative state most of the time. As a result, the model could more precisely pinpoint the psychological traits of students in the above two states and determine if they are more likely to experience depression. In contrast, the possible depression level is in the middle of the above two conditions, and the psychological and affective cognition characteristics of students in this condition are vague and not easy to identify, thus leading the model to be prone to misjudgment in the assessment, which affects the accuracy of the assessment. Overall, the average assessment accuracy of the algorithm proposed in this paper reached 85.8%, indicating that the model has strong discriminative power in determining whether students have depressive tendencies and can accurately detect students in abnormal psychological states, which has some practical application value.

The article "A Novel Adaptive Affective Cognition Analysis Model for College Students Using a Deep Convolution Neural Network and Deep Features" was published in 2022. Journal: Comput Intell Neurosci.

Compared with the traditional assessment methods based on a single data source, this study uses the multisource student behavior data recorded in the smart campus platform as the basis and uses a deep learning algorithm to extract the deep semantic knowledge and psychological and affective cognition characteristics of students contained in these data, which is more advantageous than traditional machine learning algorithms in terms of assessment accuracy. In real life, this research also helps to achieve rapid positioning and continuous tracking of students' affective cognition status. In this way, problems can be discovered in time, and active push warnings can be provided for school teachers and administrators to realize the development of students' psychological problems from “passive management” to “active prevention”.

## 6. Conclusions

This work seeks to combine deep learning technology to investigate a novel affective cognition analysis technique for college students associated with the smart campus in order to realize intelligent assessment and early warning of college students' mental health concerns. Most of the existing related research studies rely on the questionnaire survey mode, which has shortcomings such as single data source, easy to hide problems, and low efficiency. These are not conducive to providing precise and real-time intervention treatment for students with the abnormal psychological state. Therefore, for the purpose of improving the comprehensiveness and accuracy of the evaluation, this research makes improvements in two aspects of data source and model training. First, relying on the intelligent campus platform of universities, this study uses multisource behavioral data to portray the affective cognition portrait of students, including access control data, learning behavior data, and network data, so as to provide more comprehensive data sources for the affective cognition assessment of college students. Second, the collected multisource data is divided into two categories: texts and images, and CNN technology is utilized for model training, which greatly improves the accuracy and efficiency of the model. The simulation results show that the novel method has better accuracy in assessing the affective cognition status of college students compared with the data of a single modality. It can accurately grasp the mental health level of students and also provides a reference for the precise and intelligent development of mental health education in colleges and universities. In the study, we use the multisource data recorded by the smart campus platform to identify the affective cognition status of students and achieve relatively satisfactory assessment results, but there are still some problems to be further solved. In this research, both image and text data from multiple-source dataset were trained using CNN models, without considering the differences between the two. In the future, it can be studied to use suitable deep neural network models for training for different modal data. For example, for images, a CNN model can be used, while for text data, an LSTM model, which is better at text analysis, can be adopted.

The article "A Novel Adaptive Affective Cognition Analysis Model for College Students Using a Deep Convolution Neural Network and Deep Features" was published in 2022. Journal: Comput Intell Neurosci.

## Figures and Tables

**Figure 1:** Scope of artificial intelligence.

**Figure 2:** Differences between deep learning and other machine learning algorithms.

**Figure 3:** Deep neural network structure.

**Figure 4:** Framework of affective cognition analysis model based on multisource data.

**Figure 5:** Multisource data system.

**Figure 6:** CNN network structure.

**Figure 7:** Assessment results of the model for different data forms.

**Figure 8:** Assessment results of different health levels.

**Table 1:** Distribution of data in multisource dataset.

Data form	Training set	Verification set	Test set
Text	2000	250	250
Images	2000	250	250

## Data Availability

The labeled dataset used to support the findings of this study is available from the corresponding author upon request.
